The article "Evaluation of Tegaran Formula ZhenHua cytotoxicity against human cancer cell lines" was retracted in 2023. Reasons: concerns about the data; concerns about the results or conclusions; concerns about the citations.

# Evaluation of Tegaran Formula ZhenHua cytotoxicity against human cancer cell lines

**DOI:** 10.1371/journal.pone.0240969

**Published:** 2020-10-21

**Authors:** Panagiotis Parsonidis, Ioanna Vlachou, Alexandra Mamagkaki, Ioannis Bouris, Vasiliki Daikopoulou, Ioannis Papasotiriou

**Affiliations:** 1 Research Genetic Cancer Centre S.A., Industrial Area of Florina, Florina, Greece; 2 Research Genetic Cancer Centre International GmbH Headquarters, Baarerstrasse, Zug, Switzerland; Luleå University of Technology, SWEDEN

## Abstract

The aim of this study is to evaluate the potential health effects of Tegaran Formula ZhenHua, a nutritional supplement used mainly by cancer patients. Its active ingredients and cytotoxicity was assessed with analytical methods and viability assays, respectively. The analytical methods consisted of dissolution, disintegration, HPLC, LC/MS, GC/MS and NMR. Cytotoxicity was assessed by MTT, SRB, CVE colorimetric viability assays in 0, 24, 48 and 72h time points. The results indicate that Tegaran Formula ZhenHua supplement did not present any cytotoxic effects due to issues related to the capsules’ solubility, distribution and identification of the active ingredient.

## Introduction

Cancer is the second leading cause of death in the world and has become an important health problem in the developed and developing countries. The number of new cases of cancer and deaths related to cancer is showing a tendency to increase per year and in the upcoming years it will be considerably larger due to the growth and aging of the population. Moreover, cancers related to risk factors such as smoking, unhealthy diet and lifestyle are on the rise and prevention should be applied in order to stop that trend [1].

Medicinal herbs have been widely used as complementary treatments for cancer. Plant-derived compounds are used in combination with conventional therapeutics in order to have a beneficial effect on the quality of life and the survival of cancer patients [2,3]. Soy beans and soy products have been extensively used as functional foods particularly in Asia. Soybeans contain isoflavones, polyphenolic chemical compounds [4], known for their protective effects on human health [5–8]. Numerous studies have shown that, when incorporated to the diet, they regulate the development of cancers, cardiovascular diseases, neurodegenerative diseases, diabetes, osteoporosis, hypertension, allergies and others [9–15]. Phytoestrogenic isoflavones are a popular alternative to estrogen therapy and usual intake of soy products is characterized safe with weak estrogenic effects [16]. Genistein, daidzein and glycitein are the most commonly studied isoflavones and are selective estrogen receptor modulators [17].

Tegaran^®^ Formula ZhenHua is a soy fermentation product that has been used as a therapeutic and nutritional supplement by cancer patients with different clinical stages. The nutritional product is made from soybeans and it contains isoflavones. The most abundant component in Formula ZhenHua is 13-methyltetradecanoic acid (13-MTD), which is a saturated branched-chain fatty acid that could effectively inhibit tumor cell growth [18].

In the present study, Tegaran^®^ Formula ZhenHua has been used to evaluate the potential cytotoxic effect it might have against human cancer cell lines. Disintegration, dissolution and solubility tests were performed in order to determine the availability and the effectiveness of the capsule. The extracts were tested with analytical methods for content identification and quantification.

## Materials and methods

### Testing material

Tegaran Formula ZhenHua capsules were purchased from Germany. The package contains 150 capsules, 123g each capsule (LOT No: L60008508). According to the information mentioned on the package, it is developed in Switzerland and produced in Germany. The distributor in Switzerland is System Biologie AG, CH-8832 Wollerau and in Germany, Gebomed, GmbH, Im Hörnle 41, 72800 Eningen. The ingredients of the product are mentioned in Table 1.

**Table 1:** Ingredient list of Tegaran Formula ZhenHua capsules.

**Ingredients**	**Daily dose (4,1g)**
Fermented soya extract (ZhenHua) in natural unprocessed form of which isoflavones account for	4,1 g
	90 mg
**Fermented soja extract (100%), filler**: magnesium stearate (herbal), capsule: hydroxypropyl methylcellulose (HPMC), gellan gum	
**Recommended dosage**: 5 capsules to be taken with water after meals during the course of the day.	
**Example dosage**: 2 capsules in the morning, 2 at midday, 1 in the evening.	
**Amino acids**	**Daily dose (4,1g)**
L-glutamic acid	18 mg
L-alanine	15 mg
L-leucine	6 mg
L-threonine	8 mg
L-arginine	11 mg
L-glycine	10 mg
L-phenylalanine	7 mg
L-serine	8 mg
L-isoleucine	7 mg
L-aspartic acid	23 mg

### Disintegration test

Disintegration Test is the first step in analyzing the pharmaceutical profile of a solid dosage form. In this study, we used three different methods in order to clarify successfully the disintegrating properties of the capsules. The disintegration apparatus is LB-2D (LeadTop, China). One capsule of Tegaran was placed in one of the baskets in each vessel (the apparatus contained two vessels). The temperature was stable at 37°C and the disintegration time was recorded continuously during the procedure. The Buffers that were used in this method were the following:

- Acidic Buffer HCl 0.1M (pH 2), Sigma-Aldrich (Louis, MO, USA).
- Neutral/Basic Phosphate Buffer Saline (PBS) 0.01 M (pH 7.4), Sigma-Aldrich (Louis, MO, USA).

Finally, an alternative approach for disintegration was followed. Initially the capsules were immersed in Acidic buffer (HCl 0.1M) for 2 hours and the immediately changed to Neutral/Basic PBS for another hour.

### Dissolution test

Dissolution Test took place in a USP Apparatus 2, Model RCZ-8B Type Medicine Dissolving Instrument (LTPM, China) Dissolution Machine. One capsule of Tegaran was placed in a rotating basket (100 cycles/min) and then immersed into a vessel containing 900 ml of buffer at 37°C±1 for 90 min. These capsules claim to be resistant to GI track fluids and soluble at small intestine area. Therefore, we used two different Buffers,

- Phosphate Buffer Saline (PBS) 0.01M/pH 6.8, Sigma-Aldrich (Louis, MO, USA).
- Phosphate Buffer Saline (PBS) 0.01M/pH 6,8—Polysorbate 80 (0,8% w/v), Sigma-Aldrich (Louis, MO, USA).

For research purposes, we also tried to dissolute the mixture of a capsule, without the shell.

### Solubility test

Acetonitrile, ethanol, methanol and dimethyl formamide were purchased from Sigma-Aldrich (Taufkirchen, Germany), tetrahydrofuran and dimethyl sulfoxide from Honeywell (Seelse, Germany) and water for injection from BIOSER (Trikala, Greece). Tests were performed by adding 1mg of Tegaran capsule content to test tubes containing 1ml of solvent and mixing by using a Stuart vortex mixer SA8 (Staffordshire, United Kingdom) for 5min at 2500rpm and an mrc sonication bath AC-150H (Essex, United Kingdom) for 5min. The quantity of each solvent was increased until final volume of 10ml and solubility was assessed visually.

### HPLC and LC-MS analysis

Genistein, glycitein and daidzein analytical standards were purchased from Sigma-Aldrich (Louis, MO, USA). Acetonitrile and water for HPLC were also purchased from Sigma-Aldrich (Taufkirchen, Germany) and glacial acetic acid was purchased from Merck KGaA (Darmstadt, Germany). LC-MS grade water and methanol were purchased from Fisher Scientific (Pittsburgh, USA) and ammonium acetate a.r. from Chem-Lab (Zedelgem, Belgium). Tegaran capsules were purchased from Germany (LOT No: L60008508) and ethanol absolute from Honeywell (Seelse, Germany).

For HPLC analysis, 10.2 mg of capsule content was weighted and dissolved in 100 ml of methanol overnight resulting in isoflavones (genistein, glycitein, daidzein) extraction (10.5 ppm). Volume of the sonicated extract was filtered through a 0.45 μm filter and analyzed further for the assay. Samples of analytical standards of genistein, glycitein and daidzein of the same concentration were also prepared in methanol.

HPLC analysis was performed using an Agilent 1260 Infinity Series equipped with a MWD detector (Agilent Technologies Inc., Richardson, TX, USA). Chromatograms were integrated and analyzed using OpenLAB Chemstation (version M8301AA, Revision C.01.07 Agilent Technologies Inc., Richardson, TX, USA).

The analysis of isoflavones was performed using a column (Zorbax Eclipse RP C18 reverse-phase, 250 mm x 4.6 mm I.D., 5 μm, Agilent, Santa Clara, CA, USA) maintained at 40°C. Mobile phase A was water, mobile phase B was acetonitrile and mobile phase C was glacial acetic acid. The mobile phases A, B and C were mixed at a ratio of 67.5: 25.0:7.5 (v/v). Flow rate was kept at 1.5 ml/min for 16min, injection volume was 10 μL and ultraviolet (UV) detection was carried out at 260 nm.

LC-MS analysis (1260 Infinity Series HPLC, 6120 Quadrupole MSD, Agilent Technologies Inc., Richardson, TX, USA) was carried out with the use of a reverse phase column, Zorbax RX-C8 (5 μm, 250 mm × 4.6 mm, Agilent Technologies, Santa Clara, CA, USA) maintained at 40°C. Chromatograms were integrated and analyzed using OpenLAB Chemstation (version M8301AA, Revision C.01.07 Agilent Technologies Inc., Richardson, TX, USA). The solvent system used was: Mobile phase A aqueous solution of 0.1% ammonium acetate and mobile phase B solution of 0.1% ammonium acetate in methanol. The separation was carried out at a 0.4 mL/min flow rate with isocratic elution of 10% solvent A and 90% solvent B for 20 min. The injection volume was 10 μL and ultraviolet (UV) detection was carried out at 260nm. Mass spectrometry analysis was performed with a 6120 Series Quadrupole System (Agilent Technologies, Santa Clara, CA, USA) equipped with an electrospray ionization source (ESI) operating in negative mode by scan analysis with a 100–1000 *m/z* scan range.

### GC-MS analysis

13-Methyltetradecanoic acid (13-MTD) was purchased from Avanti POLAR LIPIDS, INC. (Alabama, USA), Tegaran capsules were purchased from Germany (LOT No: L60008508) and ethanol absolute from Honeywell (Seelse, Germany).

0.2mg of 13-MTD were dissolved in 1ml of ethanol (200ppm) and 1mg of Tegaran powder was extracted overnight with 1ml of ethanol. The final solution (1000ppm) was filtered through a nylon filter (d = 13mm, 0.45μm) and added to a vial for analysis.

The qualitative analysis of Tegaran was performed on a GC-MS spectrometer, Agilent GC 7890B, MSD 5977B series and Agilent G4513A injector (Agilent Technologies Inc., Richardson, TX, USA). Chromatograms were integrated and analyzed using Mass Hunter Qualitative Analysis (version B.07.00, Agilent Technologies Inc., Richardson, TX, USA). Analysis was performed by using a capillary column (Agilent CP7462, 30m x 0.25mm I.D. x 0.15μm, Agilent, Santa Clara, CA, USA). The carrier gas was helium with a flow rate set at 10ml/min and the inlet temperature was kept at 260°C with a split ratio of 30:1. The oven temperature program was 140°C for 5min, raised to 240°C at 4°C/min, the injection volume was 1μL and the transfer line temperature was 280°C. The solvent delay was set to 8min and the MSD acquisition mode was scan with a 40-400amu range.

### NMR analysis

^1^H-NMR and DOSY spectra were obtained using a Bruker Avance spectrometer at 400 MHz proton frequency (AV-III-HD, 400, Rheinstetten, Germany). Four samples were prepared by adding 5mg of Tegaran powder to 0.5ml of MeOD, DMSO-d_6_, D_2_O and D_2_O pH = 14. The NMR experiments were performed with the following parameters: Pulse angle, 30°; pulse width, 41.6 μs; data points 96152; and number of scans, 64; acquisition time (AQ), 3.999 s; spectral width, 12019.23 Hz. A line-broadening factor of 0.1 Hz was applied to FIDs before Fourier transformation, and the repetition delay was 60 s. All chemical shifts were reported in parts per million (ppm) relative to the deuterated solvents used. No solvent signal suppression and no reference standard was used. All spectra were automatically corrected for phase and baseline distortions using TOPSPIN (version 3.5pl5, Bruker Biospin, Spring, TX, USA). For DOSY ^1^H NMR, stimulated echo bipolar gradient pulse experiments were used with a pulse delay of 5 ms after each gradient, a pulse-field gradient length of 1 ms and a diffusion delay of 100 ms.

All data were processed with TOPSPIN (version 3.5pl5, Bruker Biospin, Spring, TX, USA) software using the maximum entropy algorithm (MaxEnt). The processing parameters were 1024 points along the Laplace spectrum diffusion axis and 20000 MaxEnt iterations. DOSY spectra are presented with chemical shift on the horizontal axis and diffusion coefficients expressed in μm^2^s^−1^ on the vertical axis.

### Cell culture

A panel of four different commercial cancer cell lines was used in the present study that were purchased from ECACC (European Collection of Authenticated Cell Cultures) (Salisbury, UK). MCF7 human breast adenocarcinoma cells (luminal type) (ECACC 86012803) were cultured in RPMI 1640 supplemented with 10% FBS, 2% L-Glutamine and 2% NEAA. MDA-MB-231 human breast adenocarcinoma cells (triple negative) (ECACC 92020424) were cultured in RPMI 1640 supplemented with 15% FBS and 2% L-Glutamine. HCT116 human colorectal carcinoma cells (ECACC 91091005) were cultured in DMEM supplemented with 10% FBS and 2% L-Glutamine. COLO699N human lung cancer cells (ECACC 93052608) were cultured in RPMI 1640 supplemented with 10% FBS and 2% L-Glutamine. RPMI 1640 Catalog#R0883 and L-glutamine Catalog#G7513-100ML were obtained from Sigma-Aldrich, Darmstadt, Germany and FBS Catalog#FB-1001/500 was obtained from BioSera, Nuaille, France. MEM Non-essential amino acids (NEAA) Catalog#M7145-100ML and DMEM (Dulbecco’s Modified Eagle Medium) Catalog#D5546 were purchased from Sigma-Aldrich, Darmstadt, Germany. Cells were cultured in a humidified incubator at 37°C and 5% CO_2_ and passaged when cells reached 80% confluence.

### Cell viability analysis

Viability was measured with MTT for cell-metabolism activity, with SRB and CVE for cellular protein content. The viable cells were seeded at a density of 2 x 10^4^ (200μl/well) in 96-well plate and incubated at 37°C and 5% CO_2_ for 24h to form a cell monolayer. After 24h of incubation, supernatant on the monolayer was aspirated and 200μl of medium and varying concentrations of the natural substances were added and incubated for 0, 24, 48 and 72h time points.

After the specific time points, 20μl of 5mg/ml MTT Catalog#M2128 (Sigma-Aldrich, Darmstadt, Germany) in PBS Catalog#P3813 (Sigma-Aldrich, Darmstadt, Germany) was added to each well and incubated for 3h at 37°C and 5% CO_2_. Supernatants were discarded and 100μl of DMSO Catalog#445103 (Carlo Erbo Reagents, Barcelona, Spain) was added and the plates were incubated for 5 min 37°C and 5% CO_2_ to solubilize the formazan crystals and absorbance was measured at 560nm and the reference wavelength was at 605nm.

For the SRB assay, at the specific time points cells were fixed by adding 100μl trichloroacetic acid Catalog#91228 (Sigma-Aldrich, Darmstadt, Germany) and with incubation at 4°C for 1h. Next, 100μl of SRB solution Catalog#341738 (Sigma-Aldrich, Darmstadt, Germany) was added in the wells for 30 min at room temperature. After that, supernatant was discarded, cells were rinsed three times with 1% glacial acetic acid Catalog#1.00063.1011 (Merck, Darmstadt, Germany) and were left to air dry. Finally, the dye was solubilized with 200μl of 10mM Tris-base pH 10.5 Catalog#T6791 (Sigma-Aldrich, Darmstadt, Germany) and absorbance was measured at 570nm and the reference wavelength was at 605nm.

For the CVE assay, at the specific time points, supernatant was removed and cells were fixed with 100μl 10% formalin for 20 min. Formalin was discarded and cells were left to air dry. Next, cells were dyed with 100μl of 0.25% aqueous crystal violet solution Catalog#HT901 (Sigma-Aldrich, Darmstadt, Germany) and left for 10 min at room temperature. Then, supernatant was discarded and cells were rinsed twice with 100μl WFI (water for injection) and were left to air dry. The dye was solubilized with 100μl of 33% glacial acetic acid Catalog#1.00063.1011 (Merck, Darmstadt, Germany) and absorbance was measured at 570nm and the reference wavelength was at 605nm.

### Statistical analysis

The experiment of cell viability determination was performed in triplicates. The average absorbance was calculated for each triplicate. Subsequently, the sample measurements were corrected for the measurement of the blank. One sample t-test was used to determine differences in the mean by comparing the treated samples with the untreated controls. P values < 0.05 were considered to indicate a statistically significant difference. Results were calculated using the Microsoft Excel 2016. The measurements from the three viability assays were used to determine the IC50 values by using the Microsoft Excel 2016.

## Results

### Acid-resistant capsules

In order to make a drug readily available to the body, it must be converted into a solution form. Thus, first it has to break down into smaller particles or granules. This step happens during disintegration. Based on the Pharmacopoeia Guidelines (USP <701>, Disintegration), this method is provided to determine if the solid pharmaceutical form disintegrated within the prescribed time. This test does not imply complete solution of the units and fragments of insoluble parts can remain on the screen of the test apparatus or adhere to the lower surface.

There is not a specified monograph in this case, thus we tested this pharmaceutical form in different ways. During the disintegration test at the acidic and the neutral/basic buffer, no disintegration was observed. The capsules remained intact, even after several minutes had passed. Because no apparent results were shown, the procedure was stopped after 30 minutes.

However, during the third way of disintegration, complete disintegration occurred. First, the acidic buffer did not affect the form of capsules and they remained intact. When the buffer changed, in almost an hour, complete disintegration occurred. This result could imply that these capsules are acid-resistant.

### The capsule and its content remain intact

In order to test the effectiveness of the capsule, its intrinsic ability to dissolve in the fluids of the GI track must be evaluated. This stage takes place prior to being absorbed into the circulation, thus it is vital to succeed. Since there is not a clear monograph for this substance, Phosphate Buffer Saline 0.01M pH 6,8 and Phosphate Buffer Saline 0.01M pH 6,8 with Polysorbate 80 0.8% were used. From the beginning, throughout and at the completion of the experiment, the capsule remained intact, without any trace of alteration.

In addition to this, the experiment was repeated using only the mixture of the capsule, since there is a chance that the acidic-resistant shell prevents the dissolution of the capsule. Even in this case, no dissolution was observed and the mixture remained undissolved at the bottom of the vessel. Consequently, no samples were collected during the experiment. In the following figure (Fig 1), the experimental observing can be seen.

**Fig 1:** Photographs during the dissolution of Tegaran capsules.

In the first two images, the remaining intact capsule is in the basket. In the bottom two images, the undissolved capsule mixture is inside the dissolution vessel.

### Slight solubility in specific solvents

The solubility was assessed visually to assist with further analysis. In non-polar solvents Tegaran is insoluble due to its ingredients (flavonoids and amino acids). Solubility was observed in several polar solvents and the results are presented in Table 2 below.

**Table 2:** Solubility test results.

SOLVENT	VOLUME	OBSERVATION
Acetonitrile	1–10 ml	insoluble
Tetrahydrofuran	1–10 ml	insoluble
Ethanol	1–10 ml	insoluble
Methanol	1–10 ml	slightly soluble
Dimethylsulfoxide	1–10 ml	slightly soluble
Dimethylformamide	1–10 ml	insoluble
Water for Injection	1–10 ml	insoluble
Water for Injection (pH = 14)	1–10 ml	slightly soluble

### Three isoflavones present in the capsule

A validated HPLC method quantified the isoflavones present in one capsule of Tegaran and the calculated quantities are presented in Table 3.

**Table 3:** Quantification results of isoflavones.

ISOFLAVONE	AMOUNT (mg)
Genistein	10.71
Glycitein	4.58
Daidzein	13.54
Total Isoflavone content	28.83

According to the HPLC chromatograms of Tegaran capsule and isoflavone analytical standards, the retention time of genistein was 6.4 min, of glycitein 4.4 min and of daidzein 3.9 min (S1 Fig).

LC-MS also confirmed the presence of the three isoflavones in the capsule by their molecular ions in the mass spectra (S2 Fig).

### Absence of 13-MTD

GC-MS analysis of 13-MTD fatty acid analytical standard showed one peak at 15.864min whose molecular weight was calculated as 242.1g/mol (S3 Fig). On the contrary, Tegaran presented several peaks, but none of them presented a mass spectrum with 13-MTD’s molecular ion, thus it can be understood that this compound is not present in the sample (S4 Fig).

### Methanol is the most appropriate solvent for downstream analysis

Tegaran was analyzed by ^1^H-NMR and DOSY-NMR in an attempt to find a solvent that could solubilize most of its contents and finally to proceed with *in vitro* cytotoxicity assays. ^1^H-NMR spectra of Tegaran were obtained in MeOD, DMSO-d_6_, D_2_O and D_2_O pH = 14 (S5–S8 Figs). MeOD and D_2_O pH = 14 spectra show peaks most of the ingredients present in the formulation in higher concentrations than DMSO-d_6_ and D_2_O. Cytotoxicity assays were performed in methanol and not in basic water because changes of pH to higher values have negative effects on all cellular processes, such as metabolism, cell growth and cell membrane permeability. In order to separate the signals of the ingredients, a DOSY NMR experiment in MeOD was performed (S9 Fig).

### Effect of 13-MTD and Tegaran on the proliferation and viability of the human cancer cell lines

According to literature 35μg/ml of 13-MTD was the optimum concentration for cytotoxicity effects, so the concentration range used was: 1.5, 3, 6, 15, 30 and 60 μg/ml. For Tegaran the concentration range used was: 0.075, 0.15, 0.3, 0.75, 1.5 and 3 mg/ml, which represent the concentrations of 13-MTD, into the total mixture (1 mg/ml of Tegaran corresponds to 20 μg/ml of active substance). The cells were incubated with each substance for 24, 48 and 72 hours. The analysis was also performed at 0 hours to set the baseline control.

Cytotoxic activity could be detected in MCF7, HCT116 and COLO699N human tumor cell lines treated with 13-MTD. The IC50 was 0.025mg/ml for MCF7 cells, 0.024mg/ml for HCT116 cells and 0.032mg/ml COLO699N cells at different time points. On the other hand, cytotoxicity of Tegaran could be detected against all human tumor cell lines but the IC50 was 0.40mg/ml for the two breast cell lines, MCF7 and MDA-MB-231, 0.003mg/ml for HCT116 cells and 0.045mg/ml for COLO699N cells. According to the results from the three viability assays (Tables 4–7) the lowest IC50 concentration was observed in HCT116 cell line with SRB assay at 24h of incubation with 13-MTD and the highest IC50 value was in MDA-MB-231 cell line with SRB assay at 48h of treatment with Tegaran.

**Table 4:** MCF7 cell line IC50 concentrations for 13-MTD and Tegaran according to CVE, SRB and MTT assay (NS- No significant).

MCF7	CVE	SRB	MTT
**13-MTD**	NS	NS	0.025 (72h) (p = 0.03)
**Tegaran**	0.66 (72h) (p = 0.03)	0.81 (72h) (p = 0.04)	0.40 (72h) (p = 0.03)

**Table 5:** MDA-MB-231 cell line IC50 concentrations for 13-MTD and Tegaran according to CVE, SRB and MTT assay (NS- No significant).

MDA-MB-231	CVE	SRB	MTT
**13-MTD**	NS	NS	NS
**Tegaran**	5.49 (48h) (p = 0.02)	6.56 (48h) (p = 0.02)	NS
	0.54 (72h) (p = 0.01)	0.40 (72h) (p = 0.03)	

**Table 6:** HCT116 cell line IC50 concentrations for 13-MTD and Tegaran according to CVE, SRB and MTT assay (NS- No significant).

HCT116	CVE	SRB	MTT
**13-MTD**	NS	0.024 (24h) (p = 0.02)	0.036 (24h) (p = 0.01)
**Tegaran**	NS	NS	0.003 (24h) (p = 0.01)

**Table 7:** COLO699N cell line IC50 concentrations for 13-MTD and Tegaran according to CVE, SRB and MTT assay (NS- No significant).

COLO699N	CVE	SRB	MTT
**13-MTD**	0.036 (48h) (p = 0.01)	0.032 (48h) (p = 0.01)	NS
**Tegaran**	1.44 (24h) (p = 0.003)	NS	0.045 (48h) (p = 0.02)
	1.57 (48h) (p = 0.03)		

In many cases, there was no effect observed to the treated samples with one of the two substances comparing to the untreated controls and as a result IC50 value could not be calculated or it was not statistically significant. The results presented to the Tables 4–7 were selected as statistically significant after the statistical analysis. On the one hand MTT assay was used for the determination of cell proliferation and on the other hand SRB and CVE assays were used for the determination of cell viability.

## Discussion

In the present study, we have investigated the effect of Tegaran^®^ Formula ZhenHua on the viability of human cancer cell lines including two human breast adenocarcinoma, one luminal type and one triple negative, one colorectal carcinoma and one lung cancer cell line. The use of soy fermentation products as dietary supplements have been used by cancer patients initially in China but nowadays in many countries [19]. Fermented products have been characterized as functional foods due to the fact that they possess bioactive or bioavailable end-compounds [20].

Soybeans contain isoflavones that have reduced bioavailability because they are conjugated to sugars and the human intestinal tract cannot absorb them. Fermentation transforms the isoflavones to the aglycone content and increases their bioavailability [19]. Our results indicated that Tegaran capsules prevent acidic hydrolysis, according to disintegration results, but during the dissolution experiments, the dissolution of the capsule in the buffer was unsuccessful. This may show that the active substances cannot be effectively absorbed and thus, have an overall effect in the human body. At this point, it is crucial to mention that even if the capsules claim to be enteric-soluble and the shell prevents its dissolution, the mixture of the capsule did not appear to be soluble in the aqueous fluids. With this said, the active compounds cannot expose their claimed activity, whatsoever. It was clear that the formulation of the capsules was not appropriate for the absorption of the capsules’ ingredients.

Different ingredients of the capsule were soluble in different solvents (isoflavones were soluble in methanol, 13-methyltetradecanoic acid was soluble in ethanol and amino acids were soluble in water), so it was difficult to have a clear view of the capsule content through analytical methods (LC-MS, GC-MS, NMR, etc.). NMR spectra in MeOD and D_2_O pH = 14 show that most of the ingredients are soluble and visible. However, all spectra were complicated due to the fact that several ingredients had overlapping peaks, including the amino acids. Amino acids were not detected as they were soluble in water and not visible in UV.

Although 13-MTD is considered to be the main ingredient of Tegaran according to the study that was performed by Zhenhua Yang [21], GC-MS analysis showed that it was either in untraceable quantity or not present in the formulation. It is considered to be a safe compound for normal human cells targeting specifically tumor cells including breast cancer MCF7 and colon carcinoma HCT116. It seems to be functional at low concentrations and there are no severe side effects or discomfort observed after the administration in animal models. The median infective dose (ID50) for MCF7 was 10μg/ml and for HCT116 it was 18.5μg/ml [22]. In the present study the IC50 values were slightly higher, 25μg/ml for MCF7 and 24μg/ml for HCT116.

According to the results, although there was a specific time point that Tegaran had a cytotoxic effect on MCF7 cell line in all three assays, there was no specific concentration to give consistent results for the rest of the cell lines. That might be attributed to low solubility issues as the undissolved material was covering the surface of cells on the plates.

Even if there was a sign of cytotoxicity, this would definitely not be attributed to 13-MTD as it was not detected by our analytical techniques, but due to the other ingredients present in the formulation. The involvement of isoflavones, genistein and daidzein, in the molecular pathways that are related to cell growth arrest and apoptosis have been explained. Induction of DNA damage by inhibition of tyrosine kinases and topoisomerase II that results in activation of p53 tumor-suppressor protein-dependent pathways [23]. Low stress induces low expression of p53 resulting in cell cycle arrest and in turn survival genes are expressed in order to repair any cell damage [24]. The effect of flavonoids on the cell cycle is depending on the concentration, the exposure time and the cancer cell line. High DNA damage leads to higher expression of p53 resulting in apoptosis to prevent passing the genetic defects to new cell generations [25].

## Conclusion

The present study shows that Tegaran, which has been used as a therapeutic supplement for cancer patients, has major formulation issues that prevents its distribution in the human body and the active ingredients that may be released result in no observed cytotoxicity against human cancer cell lines.

## Supporting information

S1 Fig HPLC chromatograms of Tegaran capsule and isoflavones analytical standards. (DOCX)

S2 Fig LC-MS Total Ion Chromatogram of Tegaran capsule in scan mode and mass spectra of the identified isoflavone peaks. (DOCX)

S3 Fig GC-MS Total Ion Chromatogram of 13-MTD fatty acid and its mass spectrum. (DOCX)

S4 Fig GC-MS Total Ion chromatogram of Tegaran and mass spectra of each peak present in the sample. (DOCX)

S5 Fig ^1^H-NMR spectrum of Tegaran in deuterated methanol. (DOCX)

S6 Fig ^1^H-NMR spectrum of Tegaran in deuterated dimethyl sulfoxide. (DOCX)

S7 Fig ^1^H-NMR spectrum of Tegaran in deuterated water. (DOCX)

S8 Fig ^1^H-NMR spectrum of Tegaran in deuterated water pH = 14. (DOCX)

S9 Fig DOSY-NMR spectrum of Tegaran in deuterated methanol. (DOCX)

S10 Fig IC50 calculation (scatter plot), y = 50, (IC50) x = 0.40 (MCF7, MTT, 72h). (DOCX)

S1 Table Absorbance Measurement and statistical analysis (MCF7, MTT, 72h). (DOCX)

S2 Table Calculation of the viability percentage of the MCF7 cell line after the treatment with Tegaran (MTT, 72h). (DOCX)

S3 Table Calculation of the cytotoxicity percentage of Tegaran against MCF7 cell line (MTT, 72h). (DOCX)
